The article "Identification of the Diagnostic Biomarker VIPR1 in Hepatocellular Carcinoma Based on Machine Learning Algorithm" was published in 2022. Journal: J Oncol.

# Identification of the Diagnostic Biomarker VIPR1 in Hepatocellular Carcinoma Based on Machine Learning Algorithm

**DOI:** 10.1155/2022/2469592

**Published:** 2022-09-15

**Authors:** Song Ge, Chen-rui Xu, Yan-ming Li, Yu-lin Zhang, Na Li, Fei-tong Wang, Liang Ding, Jian Niu

**Affiliations:** ^1^Department of General Surgery, The Affiliated Hospital of Xuzhou Medical University, Xuzhou, China; ^2^Institute of Digestive Diseases, Xuzhou Medical University, Xuzhou, China; ^3^Department of Oncology, Xuzhou Central Hospital, Xuzhou, China

## Abstract

The purpose of this study was to identify the potential diagnostic biomarkers in hepatocellular carcinoma (HCC) by machine learning (ML) and to explore the significance of immune cell infiltration in HCC. From GEO datasets, the microarray datasets of HCC patients were obtained and downloaded. Differentially expressed genes (DEGs) were screened from five datasets of GSE57957, GSE84402, GSE112790, GSE113996, and GSE121248, totalling 125 normal liver tissues and 326 HCC tissues. In order to find the diagnostic indicators of HCC, the LASSO regression and the SVM-RFE algorithms were utilized. The prognostic value of VIPR1 was analyzed. Finally, the difference of immune cell infiltration between HCC tissues and normal liver tissues was evaluated by CIBERSORT algorithm. In this study, a total of 232 DEGs were identified in 125 normal liver tissues and 326 HCC tissues. 11 diagnostic markers were identified by LASSO regression and SVM-RFE algorithms. FCN2, ECM1, VIRP1, IGFALS, and ASPG genes with AUC>0.85 were regarded as candidate biomarkers with high diagnostic value, and the above results were verified in GSE36376. Survival analyses showed that VIPR1 and IGFALS were significantly correlated with the OS, while ASPG, ECM1, and FCN2 had no statistical significance with the OS. Multivariate assays indicated that VIPR1 gene could be used as an independent prognostic factor for HCC, while FCN2, ECM1, IGFALS, and ASPG could not be used as independent prognostic factors for HCC. Immune cell infiltration analyses showed that the expression of VIPR1 in HCC was positively correlated with the levels of several immune cells. Overall, VIPR1 gene can be used as a diagnostic feature marker of HCC and may be a potential target for the diagnosis and treatment of liver cancer in the future.

## 1. Introduction

Liver cancer is the sixth most common cancer in the world and the fourth leading cause of cancer death [1]. The main risk factors for primary liver cancer are viral infection (mainly HBV and HCV), alcoholic and nonalcoholic steatohepatitis, aflatoxin and parasitic infections, etc. Hepatocellular carcinoma (HCC) is the most common primary liver malignancy, accounting for about 75% of all liver cancers [2, 3]. Although some progresses have been made in the diagnosis and treatments of HCC [4], more than 70%-80% of patients are still diagnosed with liver cancer at a later stage, and more than 15% of patients have extrahepatic spread at the time of diagnosis, which leads to a poor outcome [5–7]. Up to now, early surgical resection of liver cancer is still the most important and effective treatment. If the tumor is detected at an early stage and surgically removed, the 5-year survival rate of patients can exceed 70% and the prognosis is better [8]. In recent decades, alpha-fetoprotein (AFP) has been applied for HCC diagnosis [9]. The abnormal level of AFP in plasma is closely related to the malignancy of liver cancer, but due to insufficient sensitivity and specificity, the effect of early diagnosis of liver cancer is still not ideal [8]. In addition, AFP also increases in other benign and malignant diseases, such as other forms of chronic liver disease, other malignant tumors, pregnancy, and so on [7, 9]. So far, specific biomarkers are still needed to improve the accurate detection of early or very early liver cancer [9]. Therefore, it is particularly important for the early diagnosis of HCC and the search for specific diagnostic markers.

In recent years, bioinformatics has developed rapidly in the field of medicine. Comprehensive bioinformatics analysis and microarray technology can be used to identify various disease-related genes and their biological functions, which is helpful to clarify the potential mechanisms of disease occurrence and development [10–13]. However, with the increase of the amount and complexity of cancer omics research data, cutting-edge technologies such as ML algorithms have been developed to deal with the increasingly large and complex cancer and other multiomics data [14, 15]. ML is a rapidly growing core subfield of artificial intelligence (AI), which enables computer technology to learn from data processing and selfimproves to predict results without explicit programming [16, 17]. There are two goals for the use of ML in medical biology: the first is to make accurate predictions in the absence of experimental data and to guide the follow-up research work through these predictions; the second is to use machine learning to deepen our understanding of medical biology [18]. Today, ML is widely recognized as a significant innovation and a pioneering method in the field of cancer multiomics data analysis. This method, which seeks to predict, diagnose, categorize, and identify biomarkers, plays a vital role in cancer research. The combination of ML and traditional bioinformatics is used to classify and identify diagnostic biomarkers of cancer, which can greatly improve the accuracy of identifying biomarkers of cancer and provide new guidance for the early diagnosis and treatment of cancer [14, 15, 19].

We downloaded several HCC microarray datasets from the GEO database for the identification of DEGs between HCC tissues and nontumor tissues and combined with ML algorithms to identify diagnosis biomarkers in DEGs for further research. Our findings suggested VIPR1 as a novel diagnostic and prognostic biomarker for HCC patients.

## 2. Materials and Methods

### 2.1. Data Download and Processing

The microarray datasets of HCC samples were downloaded from the GEO database (http://www.ncbi.nlm.nih.gov). After screening, GSE57957, GSE84402, GSE112790, GSE113996, GSE121248, and GSE36376 datasets were included in our research (Table 1). Among them, GSE57957 included 39 normal specimens and 39 liver cancer specimens, and the platform was from GPL10558; GSE84402 included 14 normal specimens and 14 liver cancer tissues, and the platform was from GPL570; GSE112790 included 15 normal specimens and 183 liver cancer tissues, and the platform was from GPL570; GSE113996 included 20 adjacent nontumor tissues and 20 liver cancer tissues, and the platform was from GPL16043; GSE121248 included 37 adjacent tissues and 70 liver cancer tissues, and the platform was from GPL570; and GSE36376 included 193 adjacent nontumor tissues and 240 liver cancer tissues, and the platform was from GPL10558. Following the instructions in the platform file, the probes were renamed to their corresponding gene terms, and the samples were separated into tumor and normal subgroups. Using the limma and SVA packages of R software, the data of GSE57957, GSE84402, GSE112790, GSE113996, and GSE121248 chips were collected into a metadata queue and corrected in batches. The experimental group consisted of 125 cases of nontumor liver tissues and 326 cases of HCC liver tissues. The verification group consisted of the GSE36376 dataset. The clinical data of HCC patients were downloaded from TCGA datasets.

### 2.2. Screening of Differentially Expressed Genes (DEGs)

Using the limma package of R software, the experimental group microarray datasets (GSE57957, GSE84402, GSE112790, GSE113996, and GSE121248) were filtered with |log FC| ≥ 1.0 and adj. *P*.val ＜ 0.05 as the thresholds to obtain DEGs. DEGs were visually drawn with heat map and volcano map through the pheatmap and ggplot2 packages of R software.

### 2.3. Functional Enrichment Analyses of DEGs

Gene Ontology (GO) is the most comprehensive gene function database at present. To explore the biological pathways and functions of related genes, KEGG can be used for biological interpretation of genomic sequences and other high-throughput data [20] and can provide additional information about how genes interact in pathways [21]. Disease Ontology (DO) integrates data about human diseases. It can be used to annotate the human genome and better show the characteristics of current human diseases to see which diseases are enriched for differential genes [22–24]. In this study, we used the clusterProfiler package to carry out GO, KEGG, and DO enrichment analyses of DEGs under the conditions of *P*-value < 0.05 and *q*-value < 0.05 to understand the biological functions and involved diseases of DEGs.

### 2.4. Gene Set Enrichment Analysis (GSEA)

Enrichment analysis using GSEA was performed in order to identify the functional items that differed most significantly between the HCC group and the control group. The GSEA enrichment analysis of the gene set was performed by the use of the clusterProfiler package of the R software. The c2.cp.kegg.v7.4.symbols.gmt gene set was chosen as the enrichment analysis gene set.

### 2.5. Identification of Diagnostic Biomarkers by LASSO Regression and SVM-RFE Algorithms

LASSO is a regression-based algorithm performed through successive shrinking operations that minimize regression coefficients to reduce the possibility of overfitting [25], thereby reducing redundancy and eliminating irrelevant genes from these analyses [26]. SVM is one of the best choices for feature selection, and it is also the most commonly used classifier for the microarray data [27]. SVM-RFE is a feature selection algorithm based on SVM [28]. In order to define the minimum classification error and avoid overfitting, the SVM-RFE algorithm is used to select the optimal genes [27, 29]. Therefore, two ML algorithms have been widely used to identify biomarkers and predict accurate and interpretable models. In our research, we used glmnet package to run LASSO regression algorithm and e1071 package to build SVM model. The value with the least cross-validation error was found as the feature markers of HCC by two ML algorithms of LASSO regression and SVM-RFE.

### 2.6. Diagnostic Value of Feature Biomarkers in HCC

The AUC value was analyzed to determine how valuable each feature gene was as a diagnostic tool. The ROC curve of each feature gene was generated from the mRNA expression data of 125 normal liver tissues and 326 HCC tissues in the experimental group by using the pROC package of R software. The accuracy of disease diagnosis was judged by AUC value, and genes with AUC > 0.85 were identified as high diagnostic value genes for further research.

### 2.7. Validation of the Differential Expression and Diagnostic Value

We used the GSE36376 dataset to verify expressions and diagnostic values of the candidate genes in order to further investigate whether the candidate genes exhibited a diagnostic significance for HCC patients.

### 2.8. The Correlations of Diagnostic Genes with OS and Clinicopathological Characteristics of Patients

Analyses of the associations of diagnostic genes with overall survival and clinicopathological characteristics of patients were performed using data from the TCGA-LIHC transcriptome as well as clinical information. Kaplan–Meier methods were applied to investigate the connections between diagnostic genes and OS, and the survminer package of the R software was applied to develop the survival curves. Both of these analyses were performed using the survival package. The univariate and multivariate assays were applied to investigate the predictive power of each diagnostic gene in HCC.

### 2.9. Evaluation of Immune Cell Infiltration

In recent years, we have come to the realization that immune cell infiltration was involved in tumor progression. The percentage of infiltrating immune cells that can be found in malignant tumors has a direct bearing on the growth and spread of tumors, as well as the development of cancer and the patients' overall prognoses [30, 31]. CIBERSORT is a bioinformatics analysis tool that can evaluate the proportions of immune cells [32]. The content of immune cell infiltration can be obtained from each sample, and then the correlations between immune cells can be analyzed. When comparing the amounts of immune cell infiltration seen in liver cancer tissues and normal liver tissues, we employed the CIBERSORT algorithm to do our comparisons. Following the exclusion of the data containing the value 0, the corrplot package of the R software was utilized to generate the pertinent heat map in order to identify correlations between the immune cells contained within the samples.

#### 2.9.1. Correlations between Diagnostic Genes and Immune Cells

Spearman rank correlation analysis was applied for the study of the relationships between the identified diagnostic markers and immune cells.

### 2.10. Statistical Analysis

All the above analyses were performed using R (4.1.3) and Perl software. Comparisons between two independent groups were analyzed by Student's *t*-test. The survival curves were calculated by the Kaplan–Meier method and the difference by the log-rank test. Moreover, the prognostic significance of the related genes was valued by Cox regression analysis. A *P* < 0.05 was considered statistically significant.

## 3. Results

### 3.1. Identification of the DEGs in HCC Datasets

In this study, the data of 125 normal liver tissues and 326 HCC tissues in the experimental group (GSE57957, GSE84402, GSE112790, GSE113996, and GSE121248) were analyzed by the use of the limma package. A total of 232 DEGs were screened, of which 58 genes were significantly upregulated and 174 genes were significantly downregulated (Figures 1(a) and 1(b)).

### 3.2. Functional Enrichment Analyses of DEGs

The biological functions of DEGs were analyzed by GO, KEGG, and DO enrichment analyses. GO enrichment analysis showed that BP of DEGs was enriched in terpenoid metabolic process, olefinic compound metabolic process, amino acid metabolic process, and small molecule catabolic process. The CC is mainly enriched in collagen-containing extracellular matrix; MF was remarkably enriched in oxidoreductase activity (Figure 2(a)). KEGG assays revealed that DEGs were mainly concentrated in retinol metabolism, cytochrome P450, chemical carcinogenesis-DNA adducts, various amino acids, and other biological metabolic activities, etc (Figure 2(b)). DO assays indicated that DEGs were involved in cancer-related diseases such as hepatitis, nonsmall cell lung carcinoma, liver cirrhosis, biliary tract cancer, cholangiocarcinoma, esophageal cancer, and so on (Figure 2(c)).

### 3.3. GSEA Enrichment Analysis

The GSEA enrichment analysis showed that complement and coagulation cascades, cytochrome P450, glycine serine and threonine metabolism, retinol metabolism, and tryptophan metabolism were highly active in normal liver tissues, while spliceosome, ribosome, proteasome, DNA replication, and cell cycle were highly active in HCC samples (Figures 3(a) and 3(b)).

### 3.4. Identification of Feature Biomarkers

We used two different ML algorithms of LASSO regression and SVM-RFE to identify potential biomarkers of HCC. 26 genes were obtained as diagnostic markers of HCC by using LASSO regression algorithm to narrow the range of DEGs (Figure 4(a)). 31 feature genes in DEGs were identified by the SVM-RFE algorithm (Figure 4(b)). Then, 11 diagnostic feature genes were obtained by intersecting the two sets of algorithms (Figure 4(c)).

### 3.5. Diagnostic Value of Feature Biomarkers in HCC

With AUC > 0.85 as the threshold, five diagnostic feature genes of FCN2, ECM1, VIPR1, IGFALS, and ASPG were identified for further research. As shown in the Figures 5(a)–5(e), the AUC values of FCN2, ECM1, VIPR1, IGFALS, and ASPG were 0.877 (95% CI 0.832-0.915), 0.870 (95% CI 0.827-0.908), 0.871 (95% CI 0.827-0.912), 0.856 (95% CI 0.811-0.899), and 0.857 (95% CI 0.813-0.898), which indicated that these five feature genes had a high diagnostic ability.

### 3.6. Validation of the Differential Expressions and Diagnostic Values

In order to obtain more reliable results, we used the GSE36376 dataset to validate our results. The results showed that the expressions of FCN2, ECM1, VIPR1, IGFALS, and ASPG were significantly downregulated in HCC (*P* < 0.05, Figures 6(a)–6(e)), and all of them had high diagnostic values (AUC > 0.85) (Figures 6(f)–6(j)).

### 3.7. The Correlations of Diagnostic Genes with OS and Clinicopathological Characteristics of Patients

First of all, we analyzed the relationships between diagnostic genes and OS of patients. The results showed that the patients with lower expression of VIPR1 and IGFALS predicted shorter OS (*P* < 0.05), while the expressions of FCN2, ECM1, and ASPG had no statistical significance with OS (Figure 7(a)). To further screen the diagnostic genes with clinical prognostic value, we analyzed the relationships between the diagnostic genes and clinicopathological characteristics of HCC patients and performed Cox regression analyses. The results showed that the lower expression of VIPR1 was associated with the poor differentiation of tumor grade classification and malignant progression of clinical stage (*P* < 0.05) (Figures 7(b) and 7(c)). Multivariate assays demonstrated that VIPR1 could be used as an independent prognostic factor for HCC (*P* < 0.05), while other diagnostic genes could not be used as independent prognostic factors for HCC (Figures 8(a)–8(e)). Finally, we identified VIPR1 as a prognostic feature biomarker gene for diagnosing HCC.

### 3.8. Evaluation of Immune Cell Infiltration

We used the CIBERSORT algorithm to calculate the proportions of immune cells in the data set of normal liver tissues and HCC tissues (Figure 9(a)). Then, the correlations between different immune cells were evaluated. The heat map showed that T cells CD8 was positively correlated with T cells CD4 memory activated (*R* = 0.35), T cells follicular helper (*R* = 0.33), and macrophages M1 (*R* = 0.30); mast cells activated was positively correlated with neutrophils (*R* = 0.33); and monocytes were positively related to dendritic cells activated and NK cells resting (*R* = 0.33). The heat map also showed that T cells CD4 memory resting was negatively correlated with T cells CD8 (*R* = −0.52) and T cells follicular helper(*R* = −0.41); mast cells activated was negatively related to mast cells resting (*R* = −0.42); and macrophages M0 was negatively correlated with macrophages M1(*R* = −0.41) (Figure 9(b)). In addition, the results of the CIBERSORT algorithm showed that the proportions of T cell regulatory(Tregs) and macrophages M0 in HCC tissues were significantly higher than that in normal tissues (*P* < 0.05), while the proportions of T cell gamma delta and macrophages M1 in HCC tissues were significantly lower than that in normal tissues (*P* < 0.05) (Figure 9(c)).

### 3.9. Correlation between VIPR1 and Immune-Infiltrating Cells

As shown, VIPR1 was positively correlated with T cell gamma delta (*R* = 0.33), T cell CD4 memory resting (*R* = 0.25), macrophages M2 (*R* = 0.2), and monocytes (*R* = 0.2) (*P* < 0.05). VIPR1 was negatively correlated with macrophages M0 (*R* = −0.41), NK cells activated (*R* = −0.29), T cell regulatory (Tregs) (*R* = −0.25), and T cells follicular helper (*R* = −0.23) (*P* < 0.05) (Figures 10 and 11).

## 4. Discussion

Despite the significant leaps forward that have been achieved in both the diagnosis and treatment of HCC, there are still a significant number of patients who are diagnosed with the disease at a more advanced stage, which results in a low rate of patient survival. AFP is the most commonly used biomarker for monitoring liver cancer, but it is still not ideal for early diagnosis of liver cancer due to its lack of sensitivity and specificity. Therefore, it is of great significance to find and study specific biomarkers for early diagnosis of HCC. In this study, we identified VIPR1 as a diagnostic feature biomarker for HCC based on a combination of the ML algorithms and traditional bioinformatics. In addition, we compared the immune cell infiltration seen in HCC tissues to that shown in normal liver tissues, and we also investigated the relationship between VIPR1 and immune cell infiltration.

We downloaded multiple HCC microarray datasets from the GEO database. 232 DEGs were identified in 125 normal liver tissues and 326 HCC tissues. The DEGs were mainly enriched in small molecule catabolic process, amino acid metabolic process, and other biological processes. Small molecules are natural compounds with relatively small molecular weight, usually referring to biological molecules with relative molecular weight less than 1000 Dalton (especially less than 400 Dalton), which can participate in many biological processes including metabolic reactions. Studying the small molecules in metabolic pathway will help people design drugs for human diseases more effectively [33]. In addition, small molecular metabolites are sensitive to endogenous and exogenous changes in the body and have great potential and value in identifying the state and phenotype of liver cancer cells [34, 35].

In cancer, malignant cells usually exhibit greater proliferative capacity and metabolism than nonmalignant cells. Due to the increased demand for growth and metabolism, an adequate supply of amino acids is necessary for cancer cells to maintain their ability to proliferate. In addition, this rapid growth and metabolism may also exhibit a vulnerability specific to cancer, which is an increase in the demand for amino acids [36, 37]. KEGG assays revealed that DEGs were mainly enriched in retinol metabolism, cytochrome P450, chemical carcinogenesis-DNA adducts, various amino acids, and other biological metabolic activities and other tumor-related pathways. DO assays suggested that DEGs were involved in various cancers and related diseases such as hepatitis, nonsmall cell lung carcinoma, liver cirrhosis, biliary tract cancer, cholangiocarcinoma, and esophageal cancer. These results suggest that DESs are activated in many cancer-related pathways.

The retinoid metabolites are involved in a wide range of biological processes, such as cell differentiation, apoptosis, and inflammatory reaction [38]. In the human body, more than 70% of retinol metabolites are stored in the liver, so changes in their content may be involved in the occurrence and development of liver cancer [39]. Cytochrome P450 (CYP450) refers to an enzyme that is abundant in the smooth endoplasmic reticulum of hepatocytes and small intestinal epithelial cells. It is involved in the synthesis of various hormones and affects hormone-related cancer, which plays an important role in the metabolism of many anticancer drugs [40]. Long-term exposure to chemical carcinogens has been linked in certain studies to the formation of DNA adducts, and experts believe that a higher concentration of these adducts may raise the risk of tumorigenesis [41].

GSEA enrichment results showed that cell cycle, DNA replication, proteasome, ribosome, and spliceosome were highly active in hepatocellular carcinoma, which may be closely related to the occurrence and development of hepatocellular carcinoma. In order to improve the diagnostic and clinical availability of HCC diagnostic markers, we used the LASSO regression algorithm to minimize regression coefficients to reduce overfitting and the SVM-RFE algorithm to generate the minimal classification error, and the two ML algorithms took the intersection to select the optimal feature genes. Then, the feature genes were analyzed for the correlations with survival prognosis and clinicopathological characteristics for further screening. Finally, VIPR1 was identified as a diagnostic feature marker of HCC.

VIPR1 is a G protein-coupled receptor that is primarily found in normal tissues and plays a vital role in a variety of physiological tasks, including the metabolism of glycogen and the regulation of the immune system [42]. According to the findings of earlier research, VIPR1 has been found to have a variety of expressions and functions, depending on the specific type of malignant tumor. For example, VIPR1 was highly expressed in breast, gastric, and colon cancers, while it was significantly low expressed in lung, liver, and other cancers [42–45]. In breast cancer, VIP or VPAC1 receptor antagonists can enhance the killing ability of chemotherapy on breast cancer cells [46]. Functionally, elevated VIPR1 expression in gastric cancer promotes the malignant progression of gastric cancer by increasing the potential of gastric cancer cells to metastasis to distant regions. Ca2+ signaling is required for the carcinogenesis and progression of gastric cancer, and activation of VIPR1 by VIP can stimulate TRPV4-mediated Ca2+ entry [43]. It has been shown that the overexpression of VIPR1 in colon cancer may be related to the activation of EGFR, which can lead to poor differentiation of colon cancer, thereby promoting cancer progression. In addition, the overexpression of VIPR1 in tumor vessels and macrophages may play an important role in cancer invasion [44]. However, the expression of VIPR1 is lower in lung cancer tissues than in adjacent tissues, and overexpression of VIPR1 in lung cancer cells can inhibit cell proliferation, invasion, and migration [45, 47]. In HCC, VIPR1 mRNA expression is negatively correlated with DNA methylation, and the transcriptional silencing of VIPR1 caused by DNA methylation may contribute to the development of HCC [42]. The above studies have shown that VIPR1 plays different roles in different cancers, which is involved in the proliferation, invasion, migration, and differentiation of cancer cells.

In recent years, it has been abundantly obvious that the infiltration of immune cells plays a key role in both the beginning and the progression of malignancies. This information was uncovered as a direct consequence of recent research. Therefore, investigating the components of immune infiltration cells in HCC and locating diagnostic biomarkers for the diagnosis of HCC could potentially impact the clinical results of HCC patients. We used a bioinformatics technique known as CIBERSOTR to determine the relative amounts of immune cell infiltration in normal liver tissues and HCC tissues so that we could further investigate the function that immune cell infiltration plays in the development of HCC. We found that the proportions of T cell regulatory (Tregs) and macrophages M0 in HCC tissues were significantly higher than that in normal tissues.

In addition, the expression of VIPR1 in HCC was positively correlated with the levels of T cell gamma delta (0.33), T cell CD4 memory resting (0.25), macrophages M2 (0.2), and monocytes (0.2), while the expression of VIPR1 was negatively correlated with macrophages M0 (0.41), NK cells activated (0.29), T cell regulatory (Tregs), and T cell follicular helper (0.23). According to the previous studies, macrophages are central players in liver fibrosis and play a bidirectional role in the regulation of matrix deposition and catabolism [48]. Monocytes can influence the tumor microenvironment through mechanisms such as induction of immune tolerance, angiogenesis, and increased tumor cell dissemination [49]. In addition, peritumoral monocytes can induce autophagy of tumor cells and promote the occurrence and development of liver cancer [50]. In hepatocellular carcinoma (HCC), T cell gamma delta shows potent antitumor efficacy and has played an important role in tumor monitoring and antitumor immunity [51]. Tregs have the ability to produce an immunosuppressive tumor environment by releasing a variety of inhibitory cytokines. Additionally, Tregs have the potential to lead to immunological dysfunction in HCC through a number of different mechanisms [52]. The above research evidence and our findings suggested that various types of immune cell infiltrations played an important role in the pathogenesis of HCC.

## 5. Conclusions

In summary, VIPR1 can be used as a diagnostic feature marker of HCC, which is distinctly related to the occurrences, developments, and immune cell infiltration of HCC. It can also be used as an independent prognostic factor of HCC and may become a potential target for the early diagnosis and treatment of HCC in the future.

## Figures and Tables

**Figure 1:** DGSs between normal liver tissues and HCC tissues in GSE57957, GSE84402, GSE112790, GSE113996, and GSE121248 datasets. (a) The volcano plots of DEGs. (b) The heat map of DEGs.

**Figure 2:** Functional enrichment analyses of DEGs. (a) GO enrichment analysis of DEGs, including BP, CC, and MF. (b) KEGG enrichment analysis of DEGs. (c) DO enrichment analysis of DEGs.

**Figure 3:** (a) GSEA enrichment analysis showed the signal pathways in normal liver tissues. (b) GSEA enrichment analysis showed the signal pathways in liver cancer tissues.

**Figure 4:** Screening process of diagnostic biomarker candidates for HCC diagnosis and several biomarkers were identified. (a) LASSO regression algorithm. (b) SVM-RFE algorithm. (c) Two ML algorithms take intersection to identify diagnostic feature genes.

**Figure 5:** ROC curves of feature genes in experimental data set. (a) FCN2. (b) ECM1. (c) VIPR1. (d) IGFALS. (e) ASPG.

**Figure 6:** Validation of diagnostic genes differential analysis and diagnostic value. (a)-(e) Differential analysis of diagnostic genes in the GSE36376 dataset. (f)-(j) ROC curves of diagnostic genes in the GSE36376 dataset.

**Figure 7:** Correlations of diagnostic genes with OS and clinicopathological characteristics. (a) The correlations of diagnostic genes with OS, (b) the correlations of diagnostic genes with tumor grade classification, and (c) the correlations of diagnostic genes with clinical stage.

**Figure 8:** Univariate and multivariate Cox regression analyses between diagnostic genes and other clinical characteristics. (a) FCN2, (b) ECM1, (c) VIPR1, (d) IGFALS, and (e) ASPG.

**Figure 9:** Evaluation of immune cell infiltration. (a) Pattern of infiltration of immune cells in normal and tumor tissues. (b) Correlations between different immune cells. (c) The difference of immune cell infiltration between normal liver tissues and HCC tissues.

**Figure 10:** Lollipop plot of the correlations between VIPR1 and infiltrating immune cells.

**Figure 11:** Scatter plot of the correlations between VIPR1 and infiltrating immune cells.

**Table 1:** Characteristics of mRNA expression profiles of HCC.

GEO series	Expression type	Platform	Sample number	
			Normal	Tumor
GSE57957	mRNA	GPL10558	39	39
GSE84402	mRNA	GPL570	14	14
GSE112790	mRNA	GPL570	15	183
GSE113996	mRNA	GPL16043	20	20
GSE121248	mRNA	GPL570	37	70
GSE3637	mRNA	GPL10558	193	240

## Data Availability

The data sets used in this study can be obtained from TCGA and GEO public databases.
